# Artificial Intelligence Algorithm-Based Ultrasound Image Segmentation Technology in the Diagnosis of Breast Cancer Axillary Lymph Node Metastasis

**DOI:** 10.1155/2021/8830260

**Published:** 2021-07-22

**Authors:** Lianhua Zhang, Zhiying Jia, Xiaoling Leng, Fucheng Ma

**Affiliations:** Department of Ultrasound, Tumor Hospital Affiliated to Xinjiang Medical University, Urumqi 830011, Xinjiang, China

## Abstract

This paper aimed to investigate the application of ultrasound image segmentation technology based on the back propagation neural network (BPNN) artificial intelligence algorithm in the diagnosis of breast cancer axillary lymph node metastasis, thereby providing a theoretical basis for clinical diagnosis. In this study, 90 breast cancer patients with axillary lymph node metastasis were selected as the research objects and rolled randomly into an experimental group and a control group. Besides, all of them were examined by ultrasound. The BPNN algorithm for the ultrasound image segmentation diagnosis method was applied to the patiens from the experimental group, while the control group was given routine ultrasound diagnosis. Thus, the value of this algorithm in ultrasonic diagnosis was compared and explored. The results showed that when the number of hidden layer nodes based on the BPNN artificial intelligence algorithm was 2, 3, 4, 5, 6, 7, and 8, the corresponding segmentation accuracy was 97.3%, 96.5%, 94.8%, 94.8%, and 94.1% in turn. Among them, the segmentation accuracy was the highest when the number of hidden layer nodes was 2. The correlation of independent variable bubble plot analysis showed that the presence or absence of capsules, the presence of crab feet or burrs in breast cancer lesions was critical influencing factors for the occurrence of axillary lymph node metastasis, and the standardized importance was 99.7% and 70.8%, respectively. Besides, the area under the two-dimensional receiver operating characteristic (ROC) curve of the BPNN artificial intelligence algorithm model classification was always greater than the area under the curve of manual segmentation, and the segmentation accuracy was 90.31%, 94.88%, 95.48%, 95.44%, and 97.65% in sequence. In addition, the segmentation specificity of different running times was higher than that of manual segmentation. In conclusion, the BPNN artificial intelligence algorithm had high accuracy, sensitivity, and specificity for ultrasound image segmentation, with a better segmentation effect. Therefore, it had a better diagnostic effect for breast cancer axillary lymph node metastasis.

## 1. Introduction

Breast cancer refers to the appearance of malignant tumors in the breast; that is, the cancer cells originate from the lobules of the ductal epithelium of the breast, and the breast cells grow out of control and are formed. Breast cancer can be divided into carcinoma in situ and invasive carcinoma based on histopathology. According to immunohistochemistry, it can also be divided into luminal A, luminal B, and triple-negative breast cancer [1]. The incidence of breast cancer is very high, ranking at the top of malignant tumors. In developed countries such as Europe and America, the incidence of breast cancer ranks first in malignant tumors [2]. According to the data released by the National Cancer Center, there were nearly 300,000 new cases of breast cancer and more than 700,000 deaths in China in 2018, with the highest incidence among women aged 45–74 years [3]. In the growth process of breast cancer, regional lymph node metastasis is prone to occur as the tumor infiltrates into the surrounding mammary gland tissues. The most common manifestation of lymph node metastasis of breast cancer is local lymph node enlargement, hardening, fusion, agglomeration, and fixation [4]. Lymph nodes, as an important filtration structure of the human body, are responsible for phagocytosis of killer cells and removal of degenerating and broken cells [5]. After cancerous transformation, the cancer cells fall off and enter the lymph node reflux, which is intercepted by the lymph nodes, so that the cancer cells stay in the lymph nodes. Due to immune and other reasons, the cancer cells cannot be killed by the lymph nodes and survive for a long time to form lymph node metastasis [6]. Generally, lymph node metastasis in superficial sites is easy to find and diagnose, while some deep lymph nodes (internal mammary lymph nodes, mediastinal lymph nodes, etc.) are not easy to find. Therefore, computed tomography (CT) and ultrasound imaging are needed for auxiliary diagnosis to improve the accuracy of diagnosis [7, 8]. However, current ultrasound is not diagnostic for some small or unformed nodules.

The back propagation neural network (BPNN) is a multilayer feedforward network trained according to the error BP algorithm, which is one of the most widely applied neural networks at present [9]. The human brain is composed of multiple neurons, and there is a certain connection between these neurons, which becomes the basic element of the brain to process information [10]. An artificial neural network is a technology that can optimize the process of calculation and judgment by imitating the structure of the human brain, to achieve functions that cannot be realized by current computers [11]. At present, BPNN is extensively used in disease auxiliary diagnosis and survival analysis, and it can be employed to screen breast cancer, cervical cancer, and diabetes [12, 13]. Medical image classification is a key point of current medical diagnosis and pattern recognition. Through image recognition and classification, the identification of diseased tissues in medical images (such as ultrasound and CT) can be realized, and information such as the location of the disease and the size and quantity of the disease can be determined [14, 15]. Studies have found that combining the texture features of medical images with BPNN, using the feature information of pixels as training samples to train the neural network, and using the trained neural network to classify and recognize images can effectively and accurately classify a given medical image [16].

To improve the accuracy of the diagnosis of breast cancer and other diseases, and to determine whether breast cancer has metastasis to lymph nodes and other parts, the clinical diagnosis is usually combined with CT, magnetic resonance, and ultrasound imaging examinations. Therefore, the BPNN algorithm model was established in this study and applied to the segmentation of ultrasound diagnostic images of patients with breast cancer axillary lymph node metastasis, to explore the application of ultrasound image segmentation technology based on artificial intelligence algorithms in the diagnosis of breast cancer axillary lymph node metastasis.

## 2. Materials and Methods

### 2.1. Research Objects and Grouping

90 breast cancer patients with axillary lymph node metastasis were selected in this study, who were treated in hospital from January 2017 to September 2020. The cases included in this study were subjected to pathological examination and ultrasound diagnostic examination before surgical treatment. In this study, all breast cancer patients were grouped randomly into two groups and underwent ultrasound examinations. After the examination, the ultrasound images of the experimental group were processed by artificial intelligent-based ultrasound image segmentation technology to diagnose breast cancer axillary lymph nodes, while the control group was directly diagnosed by routine ultrasound images. The study had been approved by the medical ethics committee of the hospital, and the patients and their family members understood the content and methods of this study and agreed to sign the corresponding informed consent.

The criteria for inclusion were defined to include patients who were diagnosed with axillary lymph node metastasis of breast cancer by previous pathological diagnosis and imaging examination, did not receive other drugs or antibiotics in the recent research, did not receive radiotherapy or chemotherapy, and were conscious and in good mental state.

The criteria for exclusion were defined to include patients who were combined with psychiatric diseases or other system diseases, suffered from tumor metastasis to other systems and tissues other than lymph nodes, had incomplete clinical data and medical history information, did not receive treatment due to personal or other factors, and had axillary lymph nodes more than 30 mm in depth.

### 2.2. Patient Ultrasound Examination

The E-ultrasound equipment (French acoustic department Aixplorer type) and SL15-4 probe were adopted in this study, and the frequency range was 4–15 MHz. Then, each patient underwent B-type grayscale, energy Doppler, and AP examinations in sequence, and the imaging parameters of each mode and the size of the sampling box remained unchanged during the study. The operation was carried out by medical staff with about 10 years of breast ultrasound examination experience, and two full-time doctors would double-blindly read the images and record the reading results. If there was a disagreement, a third experienced physician would interpret the results.

### 2.3. BPNN Artificial Intelligence Algorithm Image Segmentation

BPNN includes three layers of feedforward network, namely, input layer, hidden layer, and output layer, and its topological structure is shown in Figure 1. The neurons of each layer are only fully connected with the neurons of the adjacent layer but not connected with the neurons of the same layer, and there is no feedback connection between the neurons of each layer, forming a feedforward neural network system with a hierarchical structure.

In the BPNN as shown in the figure, the input layer and the output layer contain *a* nodes and *b* nodes, so the neural network can be regarded as a mapping from an *a*-dimensional vector to *a b*-dimensional vector. According to the nodes of the input layer and output layer, the number of nodes in the hidden layer of the network can be calculated as follows:

(1) $$\begin{array}{c} N=\sqrt{a+b}+C. \end{array}$$

In (1), *N* stands for the number of nodes in the hidden layer, *a* means the number of nodes in the input layer, *b* represents the number of nodes in the output layer, and *C* expresses the adjustment constant. The relationship between the output and input of the artificial neural network can be expressed as follows:

(2) $$\begin{array}{c} {\text{net}}_{u}=\sum_{v=1}^{b}Q_{uv}I_{v}-p, \end{array}$$

(3) $$\begin{array}{c} O_{u}=A\left({\text{net}}_{u}\right). \end{array}$$

In (2) and (3), *I*, *Q*, *p*, *O*, and *A* stand for the input signal from the neuron, the connection weight between neurons, the bias, the output of the neuron, and the activation function in turn, so the net is the net activation. Besides, *v* and *u* represent the number of neurons. Suppose there is an *a*-layer neural network and the sample *m* is added to the input layer, so the input sum of *u* neurons at layer *n* is *S*_*u*_^*n*^ and the output is *I*_*u*_^*n*^. The weight coefficient from the *v*-th neuron in the *n* − 1-th layer to the *n*-th neuron in the *n* − 1-th layer is *Q*_*uv*_, and the excitation function of each neuron is *A*:

(4) $$\begin{array}{c} A\left(m\right)=\frac{1}{1+\exp\left(-m\right)}. \end{array}$$

In the above equation, *m* represents the number of samples. The relationship between each variable can be expressed as a mathematical relationship in

(5) $$\begin{array}{c} m_{u}^{n}=A\left(S_{u}^{n}\right), \end{array}$$

(6) $$\begin{array}{c} S_{u}^{n}=\sum_{v}Q_{uv}m_{v}^{n-1}. \end{array}$$

The BPNN algorithm is divided into two steps: forward propagation and back propagation. The forward propagation is carried out in the order of the input layer-hidden layer-output layer. What is more, the actual output is compared with the expected output. If there is a difference between the two, it enters BP. Then, the error signal will be transmitted back in reverse according to the forward propagation path, and the weight coefficient of each neuron in each hidden layer will be modified to minimize the error signal. The propagation process is shown in Figure 2.

The BP error function is defined as (7), and its gradient is determined as (8):

(7) $$\begin{array}{c} r=\frac{1}{2}{\sum_{u}\left(I_{u}^{a}-O_{u}\right)}^{2}, \end{array}$$

(8) $$\begin{array}{c} \frac{\partial r}{\partial Q_{uv}}=\frac{\partial r}{\partial S_{u}^{n}}\cdot \frac{\partial S_{u}^{n}}{\partial Q_{uv}}. \end{array}$$

Among them, *r* represents the BP error, *Q* indicates the weight, and *Ou* means the output of the neuron *u*. If *d*_*u*_^*n*^=∂*r*/∂*S*_*u*_^*n*^, the following equation can be obtained:

(9) $$\begin{array}{c} \frac{\partial r}{\partial S_{u}^{n}}=\frac{\partial r}{\partial I_{u}^{n}}\cdot \frac{\partial I_{u}^{n}}{\partial S_{u}^{n}}. \end{array}$$

In (9), *I*_*u*_ represents the input of neuron *u*, *S*_*u*_^*n*^ stands for the total input of neuron *u* in the *n*-th layer, and ∂*I*_*u*_^*n*^/∂*S*_*u*_^*n*^=*A*′(*S*_*u*_^*n*^); *A*′(*S*_*u*_^*n*^)=(1/1+exp(−*S*_*u*_^*n*^))′; (1/1+exp(−*S*_*u*_^*n*^))′=*I*_*u*_^*n*^(1 − *I*_*u*_^*n*^). Besides, ∂*r*/∂*I*_*u*_^*n*^=∂*r*/∂*I*_*u*_^*a*^ and ∂*r*/∂*I*_*u*_^*a*^=(*I*_*u*_^*a*^ − *O*_*u*_) when *n* = *a*, but ∂*r*/∂*I*_*u*_^*n*^=∑_1_(∂*r*/∂*S*_1_^*n*+1^)*·*(∂*S*_1_^*n*+1^/∂*I*_*u*_^*a*^) and ∑_1_(∂*r*/∂*S*_1_^*n*+1^)*·*(∂*S*_1_^*n*+1^/∂*I*_*u*_^*a*^)=∑_1_*Q*_*Iu*_*·d*_1_^*n*+1^ when *n* < *a*.

Therefore, the neural network weight modification equation is presented in

(10) $$\begin{array}{c} \Delta Q_{uv}\left(t+1\right)=\alpha \Delta Q_{uv}\left(t\right)-\theta \cdot d_{1}^{n}\cdot I_{v}^{n-1}. \end{array}$$

If *I*_*u*_^*n*^=*e*, *d*_1_^*n*^=*I*_*u*_^*n*^(1 − *I*_*u*_^*n*^)∑*Q*_*Iu*_*·d*_1_^*n*+1^. In addition, *Q*, *I*, *r*, and *a* stand for the weight, the input, the propagation error, and the number of nodes in the input layer, respectively.

### 2.4. Evaluation Indicators

In this study, specificity (Spe), sensitivity (Sen), and accuracy (Acc) were employed to quantitatively evaluate the performance of the processing model. The calculation method of Spe was displayed in (11), which represented the proportion of correctly classified samples in all negative samples; the calculation method of Sen is shown in (12), which indicated the proportion of samples that were correctly classified in all positive samples; Acc could be calculated in (13), which represented the proportion of training positive samples in all predicted positive samples:

(11) $$\begin{array}{c} \text{Spe}=\frac{\text{TN}}{\text{TN}+\text{FP}}, \end{array}$$

(12) $$\begin{array}{c} \text{Sen}=\frac{\text{TP}}{\text{TP}+\text{FN}}, \end{array}$$

(13) $$\begin{array}{c} \text{Acc}=\frac{\text{TN}+\text{TP}}{\text{TN}+\text{TP}+\text{FP}+\text{FN}}. \end{array}$$

In the above equations, TN stood for the number of true negative samples, representing the number of actual negative samples classified as negative samples; FP was the number of false positive samples, expressing the number of actual negative samples classified as true samples; TP was the number of true samples, which represented the number of actual positive samples classified as true samples; FN meant the number of false negative samples, which expressed the number of actual positive samples classified into negative samples.

BPNN has three or more layers of the forward network, the number of layers mainly depends on the number of hidden layers, and any continuous function in a closed interval can be approached by a single hidden layer of BPNN. Therefore, a three-layer BPNN can complete the mapping from the *n* dimension to the *m* dimension. In a neural network, the determination of the number of hidden layer nodes is the most important link in the determination of the whole network structure. In this study, through a simple cross-validation method, the number of potential hidden layer nodes was tested from 2 to 8, to explore the influence of neural network structure of different hidden layer node number models on the segmentation accuracy of ultrasonic images.

### 2.5. Statistical Methods

The data processing in this study was analyzed by SPSS 19.0 version statistical software, the measurement data were expressed as the mean ± standard deviation (¯*x* ± *s*), and the count data were represented by the percentage (%). The analysis of variance was used for pairwise comparison. In addition, *P* < 0.05 indicated that the difference was statistically substantial.

## 3. Results

### 3.1. Ultrasound Images of Breast Cancer Axillary Lymph Node Metastasis

Figure 3 shows the ultrasonographic images of breast cancer patients with axillary lymph node metastasis. It was found that most lymph nodes of breast cancer patients were oval, and the ultrasonographic images included the outer hypoechoic cortex and the inner hyperechoic medulla. In Figures 3(d)–3(f), the structure of lymph node metastasis was destroyed, the skin and medulla structure were not clear, and the local cortex showed obvious uneven thickening, with localized protrusion and eccentricity thickening (the thickness of one end of the cortex was about twice that of the other end).

### 3.2. Diagnosis Accuracy Rate of Different Hidden Layer Nodes

The average accuracy of different hidden layer nodes was compared, and the results are presented in Figure 4. When the number of hidden layer nodes was 2, 3, 4, 5, 6, 7, and 8, the corresponding segmentation accuracy was 97.3%, 96.5%, 94.8%, 94.8%, and 94.1%, respectively. In other words, the segmentation accuracy was the highest (97.3%) when the number of nodes in the hidden layer is 2. With the increase of the number of nodes in the hidden layer, the segmentation accuracy of ultrasonic images decreased continuously.

### 3.3. Analysis of the Importance of Ultrasound Manifestations and Pathological Results of Independent Variables

Figure 5 indicates the pathological findings of axillary lymph node metastasis in patients with breast cancer. The ultrasound imaging data of the patients included in the study were analyzed, and the pathological examination results of breast cancer patients with axillary lymph node metastasis were classified, including morphological regularity, echo intensity, and presence or absence of sand-like microcalcification. Different imaging features were used as independent variables, patient age was used as a covariate, and the occurrence of axillary lymph node metastasis was used as a dependent variable to establish an analysis model. According to the correlation analysis of the independent variable bubble chart (Figure 5), the presence or absence of the capsule and the presence or absence of crab feet or burrs in breast cancer lesions were important influencing factors for the occurrence of axillary lymph node metastasis, and the standardization importance was 99.7% and 70.8%, respectively.

### 3.4. Sensitivity Curve of the Algorithm Model

To determine the classification sensitivity of the BPNN model in this study, a two-dimensional ROC was drawn, and the area under the ROC curves segmented by artificial segmentation and the BPNN artificial intelligence algorithm were compared. Thus, there was an investigation on the sensitivity of the BPNN artificial intelligence algorithm to segment ultrasound images, and the results are shown in Figure 6. The area under the ROC curve classified by the BPNN artificial intelligence algorithm model was always larger than the area under the artificial segmentation curve. In other words, the BPNN artificial intelligence algorithm model had a better classification effect and high sensitivity.

### 3.5. Analysis of the Accuracy of the Algorithm Model

Figure 7 shows the accuracy analysis results of ultrasound images of breast cancer axillary lymph node metastasis by artificial segmentation and BPNN artificial intelligence algorithm. When the running times were 1, 2, 3, 4, and 5, the segmentation accuracy of the BPNN artificial intelligence algorithm model was 90.12%, 91.28%, 94.35%, 93.21%, and 95.43%, respectively. Furthermore, the accuracy was high.

### 3.6. Analysis of the Specificity of the Algorithm Model

The accuracy results of ultrasound images of breast cancer axillary lymph node metastasis by artificial segmentation and BPNN artificial intelligence algorithm were analyzed, as shown in Figure 8. When the number of running times was 1, 2, 3, 4, and 5, the segmentation accuracy of the BPNN artificial intelligence algorithm model was 90.31%, 94.88%, 95.48%, 95.44%, and 97.65% in turn. Therefore, the segmentation specificity of different running times was all higher than the manual segmentation method.

## 4. Discussion

The lymphatic system is a crucial defensive system in the human body, which is distributed throughout the body, and the lymph nodes are an important part of the lymphatic system, mostly located in the armpits, groin, neck, etc. [17]. The presence or absence of breast cancer with axillary lymph node metastasis not only affects the choice of treatment options, but also has important implications for prognostic evaluation. Chien et al. [18] found that about 60% of breast cancer patients had regional lymph node metastasis (axillary, internal breast, and supraclavicular), and 40% of them had axillary lymph node metastasis, and most of them were sentinel lymph node metastasis. What is more, the 10-year survival rate of patients without axillary lymph node metastasis was higher than the rate of patients with axillary lymph node metastasis. Therefore, the noninvasive examination of axillary lymph node metastasis for early diagnosis has become a critical issue worthy of attention in clinical work. The scope of breast cancer surgery includes breast and axillary lymph nodes [19], and breast surgery includes enlarged tumor resection and total mastectomy. Sentinel lymph node biopsy and axillary lymph node dissection are available for axillary lymph nodes, and axillary lymph node status is required except for carcinoma in situ. The choice of surgical procedure should consider the clinical stage of the tumor and the patient's physical condition. In this study, patients with breast cancer axillary lymph node metastasis were selected as the research objects. The patients were diagnosed by ultrasound and the images were segmented by artificial segmentation and BPNN artificial intelligence algorithm, and the accuracy, specificity, and sensitivity of the two segmentation methods were compared, so as to investigate the application of ultrasonic image segmentation technology based on artificial intelligence algorithm in the diagnosis of breast cancer axillary lymph node metastasis. As a result, when the number of hidden layer nodes was 2, 3, 4, 5, 6, 7, and 8, the corresponding segmentation accuracy rates were 97.3%, 96.5%, 94.8%, 94.8%, and 94.1%, respectively. It showed that the segmentation accuracy rate was the highest when the number of hidden layer nodes was 2 in the algorithm model constructed by this research, so the optimal number of hidden layer nodes for this model was 2. According to the correlation analysis of the independent variable bubble chart, the presence or absence of the capsule and the presence or absence of crab feet or burrs in breast cancer lesions were important influencing factors for the occurrence of axillary lymph node metastasis, and the standardization importance was 99.7% and 70.8%, respectively. It indicated that tumor metastasis was affected greatly by the presence or absence of the capsule and the presence or absence of crab feet or burrs in the tumor lesion. The area under the ROC curve classified by the BPNN artificial intelligence algorithm model was always greater than the area under the artificial segmentation curve, namely, the BPNN artificial intelligence algorithm model had a better classification effect and high sensitivity; the algorithm's segmentation accuracy was 90.31%, 94.88%, 95.48%, 95.44%, and 97.65% in turn, suggesting that the segmentation specificity after different running times was higher than the manual segmentation method. This was similar to the research findings of Yang et al. [20], which disclosed that the BPNN artificial intelligence algorithm had high accuracy, sensitivity, and specificity for ultrasound image segmentation, and the segmentation effect was better. Moreover, it also had a better diagnostic effect for breast cancer axillary lymph node metastasis.

## 5. Conclusion

In this study, the BPNN artificial intelligence algorithm model was constructed and applied to the ultrasound images of breast cancer lymph node metastasis, and the images were segmented, so as to explore its application value in the diagnosis of breast cancer axillary lymph node metastasis. The results showed that the BPNN artificial intelligence algorithm had high accuracy, sensitivity, and specificity for ultrasound image segmentation, with better segmentation effect, which also had a better diagnostic effect for breast cancer axillary lymph node metastasis. However, the selected case samples in this study are small, which may have a certain impact on the experimental results. In addition, it lacks a comparison with other intelligent algorithm segmentation effects, and the representativeness is low. Therefore, the sample size will be increased in subsequent experiments, thereby further analyzing the application of ultrasound segmentation technology based on artificial intelligence algorithm in the diagnosis of breast cancer axillary lymph node metastasis. All in all, the results of this study can provide data support and theoretical basis for clinical diagnosis of breast cancer lymph node metastasis and other diseases.

## Figures and Tables

**Figure 1:** The structure of BPNN.

**Figure 2:** BPNN workflow chart.

**Figure 3:** Ultrasound images of breast cancer axillary lymph node metastasis (note: (a–c) were left axillary lymph nodes; (d–f) were right axillary lymph nodes).

**Figure 4:** The average correct rate of different hidden layer nodes.

**Figure 5:** Comparison of the importance of the pathological results of independent variables (the independent variables 1–10 in the above figures represented the tumor shape, boundary, capsule, crab feet or burrs, internal echo, whether the echo was uniform, posterior echo, sand-like microcalcification, blood flow, and axillary lymph nodes).

**Figure 6:** ROC curve of BPNN.

**Figure 7:** Algorithm segmentation accuracy analysis.

**Figure 8:** Algorithm segmentation specificity analysis.

## Data Availability

No data were used to support this study.
